RETRACTED

# Efficacy of Chinese Medicine Injection for Cardiotoxic Injury of Anthracycline Chemotherapy Drugs: A Network Meta-Analysis of Randomized Controlled Trials

**DOI:** 10.1155/2022/5800575

**Published:** 2022-03-31

**Authors:** Mingxuan Li, Hongdian Li, Hongxu Liu, Xiaolei Lai, Wenlong Xing

**Affiliations:** ^1^Beijing University of Chinese Medicine, Beijing, China; ^2^Beijing Hospital of Traditional Chinese Medicine, Capital Medical University, Beijing, China

## Abstract

**Background:**

Chinese medicine injections (CMIs) are widely used in the prevention and treatment of cardiotoxicity caused by anthracycline chemotherapeutic drugs. However, it is uncertain that CMIs are more effective in combating the cardiotoxicity of anthracyclines. The aim of this Network Meta-analysis (NMA) was to compare the treatment effects of various CMIs in order to determine the best CMI for the prevention and treatment of cardiac damage from anthracyclines.

**Methods:**

The Chinese Journal Full Text Database (CNKI), Wanfang Database, Chinese Science and Technology Journal Full Text Database (VIP), Chinese Biomedical Literature Database (CBM), PubMed, Web of Science, and Cochrane Library databases were searched to screen randomized controlled trials (RCTs) of CMIs against cardiotoxicity of anthracycline-based chemotherapeutic drugs. The search time frame was all from the establishment of the database to October 1, 2021. After independent screening of the literature, extraction of information and evaluation of the risk of bias of the included studies by two evaluators, mesh meta-analysis was performed using RevMan 5.3, Stata 15.1, and ADDIS 1.16.8 software.

**Results:**

A total of 33 studies including 2783 patients, including 1410 cases in the experimental group and 1373 cases in the control group were included, and six CMIs were extracted, namely, Shenfu injection, Shenmai injection, Shenqi Fuzheng injection, Shengmai injection, Xinmailong injection, and Haungqi injection. The results of the reticulated meta-analysis showed that in terms of ST-T segment (ECG change) change rate, Haungqi injection, Shenfu injection, and Xinmailong injection were superior. In terms of lowering CK-MB, Huangqi Injection and Shenqi Fuzheng injection were superior. In terms of improving Left ventricular ejection fraction (LVEF), Shenfu injection, Huangqi Injection, and Shengmai injection were more effective than other injections. In terms of improving LVEDD, Shengmai injection, Huangqi Injection, and Xinmailong injection have advantages.

**Conclusion:**

The six CMIs included in this study are effective against cardiotoxicity caused by anthracycline-based chemotherapeutic agents. Huangqi Injection and Shenfu injection are both superior in improving various outcome indicators. There is still a need for larger, high-quality randomized controlled trials (RCTs) to compare the various CMIs in a more refined way.

RETRACTED

## 1. Introduction

Fifty years on from its discovery, anthracycline anti-tumor and cardiotoxic mechanisms alike continue to evoke considerable interest in basic science and clinical trials research [1]. They are widely used in the chemotherapy of many malignancies, such as lymphoma and breast cancer, and are the basic drugs in commonly used oncologic chemotherapy regimens. One of the common adverse effects of anthracycline-based chemotherapeutic agents is cardiotoxicity, a toxic reaction caused by multiple molecular processes focused on altered myocardial cell function and cytopathic death [2]. Anthracycline cardiotoxicity may be acute or chronic depending on the onset of the first symptomatic manifestations [3]. As the dose of anthracyclines increases, the cumulative toxic effect on the heart becomes greater, which in turn affects the prognosis of oncology patients [4]; therefore, prevention of anthracycline-induced cardiotoxicity cannot be ignored. Dexrazoxane represents the only pharmacological therapy approved by both the US Food and Drug Administration and the European Medicines Agency (EMA) as a cardioprotective agent during treatment with anthracyclines [5, 6]. However, dexrazoxane is for the prevention of anthracycline cardiotoxicity and not for the treatment of heart failure and cardiomyopathy caused by anthracyclines.

The literature reports that Chinese medicine injections (CMIs) neither affect the antitumor effects of anthracyclines nor reduce the incidence of cardiotoxicity [3]. Ohnishi and Takeda [7] analyzed a variety of Chinese herbal ingredients and found that CMIs can help counteract the cardiotoxicity produced by anthracyclines by reducing nitric oxide production and producing calcium antagonism to inhibit cardiomyocyte apoptosis. CMIs has a clearer composition and is easier to standardize than, for example, herbal tonics and acupuncture treatments. Several clinical trials have shown that CMIs are effective in combating cardiac damage caused by anthracyclines [8–14].

A meta-analysis of dozens of RCTs comparing the efficacy of CMIs for the prevention and treatment of anthracycline-induced cardiotoxicity has been published [15–17] There are no head-to-head RCTs on the efficacy of these CMIs, and most doctors are not able to select the appropriate CMI based on the unique “diagnosis and treatment” approach of Chinese medicine. Therefore, We adopted a Bayesian network Meta-analysis to compare the effects of six commonly used CMIs (Table 1) on cardiac damage from anthracycline-based chemotherapy drugs and rank their benefits in the hope of finding one or more of the more effective CMIs for clinicians.

RETRACTED

## 2. Methods

### 2.1. Study Registering and Reportin

This programme is based on the Preferred Reporting Items for Systematic Reviews and Meta-Analyses Programme (PRISMA-P) [18]. The PRISMA Extension Statement is used to ensure that all aspects of the method and results are reported [19].

### 2.2. Eligibility Criteria

The Population-Intervention-Comparators-Outcomes-Study design (PICOS) framework was adopted as the eligibility criteria for the review as following.

#### 2.2.1. Study Design

Randomized controlled trials (RCTs) on CMIs for the treatment of cardiotoxicity of anthracycline-based chemotherapeutic agents, unrestricted, blind method, language.

#### 2.2.2. Population

Patients with various types of tumors without serious basic heart disease who were treated with regular anthracycline chemotherapy (e.g., Adriamycin, Epirubicin, Daunorubicin, Aclacinomycin). Diagnostic criteria must be in accordance with the accepted diagnostic criteria for each type of tumor relevant to the study at the time of publication; patients are enrolled regardless of age, gender, race, geography, disease duration, and ethnicity.

#### 2.2.3. Interventions/Comparators

We conducted a preliminary analysis of the literature related to the treatment of cardiac damage from anthracyclines and found that the six most commonly used CMIs are for cardiac damage from anthracyclines. The six CMIs are the following: Shenfu injection, Shenmai injection, Shenqi fuzheng injection, Shengmai injection, Xinmailong injection, and Huang qi injection. For the purpose of data analysis, we defined conventional treatment as the administration of supportive, antiemetic, and symptomatic treatments. A comparison of those eligible is as follows: Control group, tumor patients whose chemotherapy regimen is based on anthracycline chemotherapy drugs, no CMIs or other cardioprotective drugs, unlimited duration, dose and route of administration, supportive, antiemetic, and symptomatic regimens may be given in conjunction with the patient's condition. Experimental group, only one CMI treatment was combined with the corresponding control group. There are no restrictions on the dose or duration of the drug.

Studies that did not meet all of these inclusion criteria were excluded. In addition, the following exclusion criteria were applied:

①repeated publications; ② personal experience summary, pure theoretical research, and animal experiment; ③ in addition to CMI, the two groups also used traditional Chinese medicine decoction, Chinese patent medicine or acupuncture and moxibustion; ④ the number of reported cases in each group was too small (<20 cases); ⑤ the treatment course of each group was too little (<7 days); ⑥ the data in the literature are incorrect or incomplete.

RETRACTED

### 2.3. Outcome Measures

From a review of clinical trials published in academic journals evaluating the cardiotoxicity of anthracyclines, we found that the commonly used evaluation parameters include cardiac biomarkers, electrocardiograms, echocardiograms, endomyocardial biopsies, etc. [20]. ECG and cardiac enzyme profile tests are now commonly used in clinical practice. The guidelines recommend using three-dimensional echocardiography (3DE), as it is more accurate in determining LVEF. [21]. Changes in cardiac function are also widely used to evaluate cardiac conditions during treatment [22–30]; therefore, the following criteria were used to determine the results. Outcome indicators Primary indicators: ①ECG ST-T segment change rate, ② creatine kinase isoenzyme (CK-MB); ssecondary indicators: ① changes in left ventricular ejection fractions (LVEF), ② left ventricular end diastolic dimension (LVEDD).

### 2.4. Data Sources and Search Strategy

Computer searches of the China Knowledge Network (CNKI), WanFang Data Knowledge Service Platform (WanFang Data), Vipshop (VIP), China Biomedical Literature Database (CBM), PubMed, Web of Science, and Cochrane Library databases were conducted, and the search time of each database was built until November 1, 2021. In addition, references to the literature were included retrospectively to supplement access to relevant literature. The search was conducted with a combination of subject terms and free terms. English search terms include “Traditional Chinese medicine injection,” “Shenfu,” “Shenmai,” “Shenqi Fuzheng,” “Shengmai,” “Xinmailong,” “Haungqi,” “anthracycline drugs,” “adriamycin,” “epirubicin,” “daunorubicin,” “doxorubicin,” “epirubicin,” “cardiotoxicity,” “heart injury,” and “random,” etc. Take PubMed as an example, the search terms and strategies are as follows:

(((((Traditional Chinese medicine [MeSH Terms]) OR (Traditional Chinese medicine [Title/Abstract])) OR (Injection [MeSH Terms])) OR (Injectable [MeSH Terms])) OR (Shenfu injection [MeSH Terms])) OR (Shenmai injection [MeSH Terms])) OR (Shenqi fuzheng injection [MeSH Terms])) OR (Shengmai injection [MeSH Terms])) OR (Xinmailong injection [MeSH Terms])) OR (Huang qi injection [MeSH Terms])) OR (Injection [Title/Abstract])) OR (Injectable [Title/Abstract])) OR (Shenfu injection [Title/Abstract])) OR (Shenmai injection [Title/Abstract])) OR (Shenqi fuzheng injection [Title/Abstract])) OR (Shengmai injection [Title/Abstract])) OR (Xinmailong injection [Title/Abstract])) OR (Huang qi injection [Title/Abstract]))) AND ((((Anthracyclines [MeSH Terms]) OR (Adriamycin [MeSH Terms])) OR (Epirubicin [MeSH Terms])) OR (Daunorubicin [MeSH Terms])) OR (Aclacinomycin [MeSH Terms])) OR (Anthracyclines [Title/Abstract])) OR (Adriamycin [Title/Abstract])) OR (Epirubicin [Title/Abstract])) OR (Daunorubicin [Title/Abstract])) OR (Aclacinomycin [Title/Abstract]))))) AND ((((Cardiotoxicity[MeSH Terms]) OR (Cardiac injury [MeSH Terms])) OR (Cardiotoxicity [Title/Abstract])) OR (Cardiac injury [Title/Abstract]))))) AND (((Randomized Controlled Trial [Title/Abstract]) OR (Controlled Clinical Trial [Title/Abstract])) OR (random)))

The search strategies of other databases have been adapted to their search rules.

RETRACTED

### 2.5. Study Selection and Data Extraction

Two investigators conducted literature screening and data extraction. After excluding duplicates, we first read the titles and abstracts of the articles and excluded those that clearly did not meet the requirements, and then read the full text of the remaining articles to clarify whether they met the inclusion criteria. Data extraction included: ①basic information: article title, first author, publication time, country/region, etc.; ② study characteristics: interventions in the trial and control groups, number of study subjects, age, and follow-up time; ③ key information required for risk of bias evaluation in the literature; and ④ outcome indicators included in the trial and control groups.

### 2.6. Quality Assessment

The research quality of RCTs was evaluated by two researchers using the tools for assessing the risk of bias recommended in Cochrane system evaluator manual 5.1 [31, 32], including the following seven aspects: random sequence generation, allocation concealment, blinding researchers and subjects, blind evaluation of research outcomes, integrity of outcome data, selective reporting of research results, and other sources of bias. Each aspect can be further classified as “low risk of bias,” “unclear risk of bias,” and “high risk of bias.” In case of disagreement, it can be decided through mutual discussion or consultation with the third researcher.

### 2.7. Statistical Analysis

Revman 5.3, Stata 15.1, and ADDIS 1.16.8 software were used for meta-analysis. The counting data are expressed by odds ratio (or) and its 95% confidence interval (CI), and the measurement data are expressed by mean difference (MD) and its 95% confidence interval (CI). Use *χ*^2^ test was used for heterogeneity analysis, and *I*^2^ was used to evaluate the heterogeneity [33]. Quality evaluation of included literature and direct comparison using RevMan 5.3. Using Stata 15.1 to draw the network relationship diagram to show the network relationship of different intervention measures. Funnel plot is drawn to identify whether there is a small sample effect evaluation. Bayesian mesh meta-analysis is carried out by using ADDIS 1.16.8. When there is a closed loop, the consistency between direct comparison and indirect comparison passes the consistency test. When the inconsistency factor (if) of consistency test is close to 0 or the odds ratio (ROR) of hypothesis test is close to 1, it is considered that there is consistency between direct and indirect evidence [34]. Four Markov chains are used to set the initial value. The number of initial update iterations of the model is 50,000 and the number of continuous update iterations is 20,000. The first 50,000 annealing times are used to eliminate the influence of the initial value. Sampling starts after 50,001 times. When the potential scale reduction factor (PSRF) tends to 1, the convergence is satisfactory [35]. Calculate the ranking results of the surface under the cumulative ranking curve (SUCRA) of each intervention measure, and finally present the results of mesh meta-analysis in tabular form to obtain the relatively best intervention measure.

RETRACTED

## 3. Results

### 3.1. Literature Screening Process and Basic Characteristics

A total of 591 literature were obtained by searching relevant databases. After excluding duplicate literature, 263 articles were obtained. By reading the titles and abstracts of the literature, 188 articles that obviously did not meet the inclusion criteria were excluded; for the remaining 75 articles, by reading the full text, 42 articles that did not meet the inclusion criteria in terms of study subjects, design types, and intervention conditions were excluded, and 33 RCTs studies were finally included [22, 23, 30, 36–59]. The literature screening process is shown in Figure 1, 33 studies were all in Chinese, with a total of 2724 patients, including 1380 in the experimental group and 1344 in the control group. Six CMIs were included, specifically: Shenqi Fuzheng Injection (11 items), Shenmai Injection (6 items), Xinmailong Injection (5 items), Shengmai Injection (4 items), Shenfu Injection (4 items), and Huangqi Injection (3 items). The basic characteristics of the included studies are shown in Table 2.

### 3.2. Evaluation of the Quality of the Included Studies

A total of 33 studies [19, 30, 33] all mentioned “random” grouping, of which 6 studies [28, 41–53, 57] used the “random number table” method for grouping, 1 study [54] used the “random number drawing method”, 1 study [45] used the “treatment order” to determine the grouping, and 1 study [56] used the “medication method” for grouping. All 33 studies did not mention allocation concealment. The data integrity of 33 studies was good. Other biases were uncertain, as shown in Figure 2.

RETRACTED

### 3.3. Results of Reticulated Meta-Analysis

#### 3.3.1. Mesh Relationship Diagram

The reticulation between the CMIs of the six included therapeutic anthracycline chemotherapeutic agents for cardiotoxicity is shown in Figure 3. The total number of arms in the 33 papers totals 66. Lines between nodes indicate direct comparative evidence between the two interventions, no lines indicate no direct comparison, indirect comparisons can be made through reticulated Meta-analysis. The thickness of the line represents the number of included studies comparing each treatment, and the circular area represents the sample size of the population using the measure.

#### 3.3.2. Consistency Testing

The seven interventions in this study did not form a closed loop and did not require consistency testing.

#### 3.3.3. ST-T Segment (ECG Change) Alteration Rates

A total of 27 studies [22–24, 27, 28, 36, 38, 40–44, 46, 47, 49, 58] were included comparing ECG ST-T segment (ECG change) alteration rates after anthracycline treatment for CMIs. The evidence plot is shown in Figure 4. The results of the Network Meta-analysis showed that the addition of Shenfu injection compared with chemotherapy only RR = 8.13, 95% CI [2.35, 31.15]; the addition of Shenmai injection compared with chemotherapy only RR = 3.20, 95% CI [1.18, 8.32]; the addition of Shenqi Fuzheng injection compared with chemotherapy only RR = 2.41, 95% CI. [1.18, 5.14]; addition of Shengmai injection compared with chemotherapy only RR = 3.53, 95% CI [1.51, 9.54]; addition of Xinmailong injection compared with chemotherapy only RR = 6.13, 95% CI. [2.38, 17.69]; addition of Hangqi injection compared with chemotherapy only RR = 6.35, 95% CI. [1.25, 42.40]. For ECG ST-T segments (ECG changes), the difference in variability was statistically significant (*P* < 0.05); see Table 3. The improvement effect of the six CMIs on ECG ST-T segment (ECG changes) variation in descending order of specific ranking (rank) was: Hangqi injection (SUCRA = 0.37), Shenfu injection (SUCRA = 0.30), Xinmailong injection (SUCRA = 0.27), Shengmai injection (SUCRA = 0.03), Shenmai injection (SUCRA = 0.03) = Shenqi Fuzheng Injection (SUCRA = 0.00), chemotherapy only (SUCRA = 0.00) shown in Figure 5.

#### 3.3.4. CK-MB

Five studies with U/L as the detection [22, 59] and six studies with ng/ml (*μ*g/L) as the detection [27, 45] were included, respectively. The evidence diagrams are shown in Figures 6 and 7 the results of the Network Meta-analysis showed that chemotherapy only was not statistically significant for the change in CK-MB values compared to the addition of CMIs (*P* > 0.05). See Table 4. The probability of improvement of CK-MB values of the four CMIs in terms of U/L in descending order (rank) was: Huangqi injection (SUCRA = 0.49), Shengmai injection (SUCRA = 0.34), Shenfu injection (SUCRA = 0.08) = Senqi Fuzheng injection (SUCRA = 0.08), chemotherapy only (SUCRA = 0.00); the probability of improvement of CK-MB values of the three CMIs in terms of ng/ml (*μ*g/L) in descending order (rank) was: Shenqi Fuzheng Injection (SUCRA = 0.71), Shenfu Injection (SUCRA = 0.19), Shenmai injection (SUCRA = 0.08), chemotherapy only (SUCRA = 0.02). Shown in Figures 8 and 9

RETRACTED

#### 3.3.5. LVEF

A total of 20 studies [23, 26, 27, 30, 36, 44–51, 53–59] were included comparing the change in LVEF values following anthracycline treatment with CMIs. The evidence diagrams are shown in Figure 10. The results of the Network Meta-analysis showed that chemotherapy only compared with the addition of Xinmailong injection MD = −2.84, 95% CI [−6.31, 0.54]; and MD = −6.45, 95% CI [−12.85, 0.29] compared with the addition of Huangqi injection, which was not statistically significant for the difference in change in LVEF values (*P* > 0.05) Shenfu Injection MD = −10.59, 95% CI [−20.19, −0.71], Shenqi Fuzheng injection MD = −4.78, 95% CI [−7.57, −1.96], Shengmai injection MD = −4.27, 95% CI [−8.37, −0.19]. Significantly better improvement in LVEF values than the control group; see Table 5. The probability of improving LVEF value after anthracycline treatment by five CMIs from high to low is as follows: Shenfu injection (SUCRA = 0.71), Huangqi injection (SUCRA = 0.21), Shengmai injection (SUCRA = 0.04), Shenqi Fuzheng injection (SUCRA = 0.03), Xinmailong injection (SUCRA = 0.01), and chemotherapy only (SUCRA = 0.00), shown in Figure 11.

#### 3.3.6. LVEDD

A total of 13 studies [36, 46, 48, 51, 53, 59] were included comparing the change in LVEDD values following anthracycline treatment with CMIs. The evidence diagrams are shown in Figure 12. The results of the Network Meta-analysis showed that there was no statistically significant difference in the change in LVEDD values between chemotherapy that only compared with the addition of Shenqi Fuzheng Injection MD = 3.62, 95% CI [−1.17, 8.32]. Shengmai injection MD = 8.18, 95% CI [4.38, 11.91], Xinmailong injection MD = 4.79, 95% CI [1.83, 7.69], Hangqi injection MD = 7.81, 95% CI [4.04, 11.58]. Significantly better improvement than control for LVEDD values; see Table 6. The probability of improving LVEDD value after anthracycline treatment by four traditional CMIs from high to low is as follows: Shengmai injection (SUCRA = 0.49), Hangqi injection (SUCRA = 0.46), Shenqi Fuzheng Injection (SUCRA = 0.03) = Xinmailong injection (SUCRA = 0.03), chemotherapy only (SUCRA = 0%). Shown in Figure 13

RETRACTED

#### 3.3.7. Assessment of Heterogeneity

The results of the heterogeneity estimates are shown in a forest plot. Our assessment showed that five studies had the least heterogeneity (*I*^2^ = 0.00%) across all comparisons on different outcomes. However, moderate-to-high heterogeneity was detected in the following comparisons.

Shenfu injection for ST-T segment (ECG change) alteration rates (46%) (Figure 14) and CK-MB (U/L) (100%) (Figure 15), Shenmai injection for CK-MB (*μ*/L) (58%) (Figure 15), Shenqi fuzheng injection for CK-MB (*μ*/L) (100%) (Figure 15), LVEF (89%) (Figure 16) and LVEDD (98%) (Figure 17), Shengmai injection for ST-T segment (ECG change) alteration rates (85%) (Figure 17) and LVEF (80%) (Figure 16), Xinmailong injection for LVEF (90%) (Figure 16) and LVEDD (60%) (Figure 17), Huang qi injection for LVEDD (75%) (Figure 17).

#### 3.3.8. Sensitivity Analysis

We differentiated by the number of cases ≥80 for sensitivity analysis and a total of 17 studies [22–25, 30, 38, 39, 41, 42, 44, 45, 50–52, 54, 56, 59] with a total of 1759 patients were included in the sensitivity analysis. The results did not show any obvious deviations from the original network meta-analysis (Tables 7–10). The results of Shenfu injection and Shengmai injection on LVEF were slightly different from the initial meta-analysis. The results of Shengmai injection、Xinmailong injection for LVEDD differ from the initial meta-analysis. No significant advantage of these CMIs over the improvement in LVEF and LVEDD with chemotherapy only.

Another sensitivity analysis was conducted to distinguish between studies with inconsistent treatment cycles. We extracted studies with ≥4 cycles of treatment for sensitivity analysis and a total of 18 studies [23, 27, 29, 37–40, 45–47, 49–51, 53–55, 58, 59] with 1568 patients were included in the sensitivity analysis. The results did not show any significant bias compared to the original network meta-analysis (Tables 11–14). ECG ST-T segment (ECG changes) variation is best treated with Xinmailong injection. Shenqi fuzheng injection best for LVEDD. Both differed only slightly from the original meta-analysis.

#### 3.3.9. The Small Sample Effect and Publication Bias

Studies with ST-T segments (ECG changes), LVEF, and LVEDD as indicators were included to produce comparison, correction funnel chart to assess small sample effects (Figures 18–20). The results show that the comparison–correction funnel plot of LVEF values shows basic symmetry and that the studies are roughly symmetrically distributed on either side of the midline, indicating that a small sample effect is less likely to exist. The symmetry of ST-T segment (ECG change) alteration rates and LVEDd value is poor, indicating that the possibility of small sample effect is greater. The reasons for this may be related to the low quality of the included studies, the small sample size, the inconsistency in the types of malignancies suffered by the baseline population, the types of CMIs used, and the different intervention regimens.

RETRACTED

## 4. Discussion

CMIs have a wide range of applications in Chinese hospitals, where they are used in the treatment of various diseases, including critical illnesses. Meta-analyses of the six CMIs included in our study were less available for the prevention and treatment of anthracycline heart damage, except for Shenfu injection and Shengmai injection. Also, no studies have been done to compare their efficacy. Several authors [60–62] have conducted Meta-analyses on the efficacy of CMIs against anthracycline cardiotoxicity and showed a highly significant benefit of CMIs in this disease. However, none of these studies distinguished between the different CMIs and simply treated all CMIs as one intervention, whereas in practice only one type of CMIs is often used for a patient. Our study pioneered a Network Meta-analysis of six CMIs for the treatment of anthracycline cardiotoxicity, can actually help doctors make more rational choices when deciding on the use of CMIs.

We decided to evaluate the included studies on four dimensions: ECG ST-T segment change rate, CK-MB, LVEF, and LVEDD, all four of which are mechanistically linked. The body surface 12-lead ECG is able to reflect various states of the subject's heart, such as the origin of the rhythm, beat frequency, myocardial ischemia or not, and electrolyte changes in the body. Elevation or depression of the ST-T segment is the best indicator of myocardial blood supply at this point in time, and regular testing can determine whether the heart has suffered any changes in myocardial blood supply over time due to injury [63]. CK-MB is a reliable index to directly reflect myocardial injury. Detecting CK-MB can reflect the changes of myocardial injury degree in different time periods [64]. LVEF is the most commonly used index to assess left ventricular systolic function and is predictive of prognosis in acute coronary syndromes, acute myocarditis, and heart failure. The left ventricular end-diastolic diameter (LVEDD) is an important tool for assessing left ventricular diastolic function, identifying patients with reduced diastolic function and helping to improve the early management and prognosis of patients with heart failure [65].

RETRACTED

This study comprehensively summarizes the efficacy of six CMIs against cardiotoxicity following anthracycline use. The results suggest that (1) Many CMIs are superior to chemotherapy only in ST-T segment (ECG change) change rate, LVEF, and LVEDD. (2) Huang qi injection, Shenfu injection, and Shengmai injection had the best effects on ST-T segment (ECG change) change rate, LVEF, and LVEDd, respectively. (3) Shenfu Injection, Shenmai Injection, Shenqi fuzheng Injection, Shengmai Injection and Huang qi Injection were not effective in improving CK-MB (U/L). Poor improvement of CK-MB (*μ*/L) with Shenfu Injection, Shenmai Injection, and Shenqi fuzheng Injection. (4) Shenfu Injection, Shenmai Injection, Shenqi fuzheng Injection, Shengmai Injection, Xinmailong Injection, and Huangqi Injection have better effect on reducing ST-T. (5) Shenfu Injection, Shenqi fuzheng Injection, Shengmai Injection, Xinmailong Injection, and Huangqi Injection are beneficial in increasing LVEF. (6) Shengmai injection, Xinmailong injection and Huang qi injection are more effective in reducing LVEDD. Combining the results of each index, Huang qi injection and Shenfu injection showed better improvement on the primary and secondary indexes and can be preferred for the treatment of patients.

Studies [66, 67] have found that the active ingredient in Shenmai Injection is a saponin compound with anti-inflammatory and anti-myocardial ischemic effects, protection and repair of cardiomyocytes and certain anti-arrhythmic effects. Shenqi fuzheng Injection can affect a variety of intracellular signaling pathways, reducing myocardial cell injury, anti-myocardial fibrosis, reversing heart failure, improving cardiac function, and inhibiting ventricular remodeling [68]. Astragaloside, the main component of Astragalus in the injection, can indirectly inhibit Na^+^-Ca^2+^ exchange by altering Na^+^-K^+^-ATPase activity, increasing Ca^2+^ to achieve cardiac strengthening, improving left ventricular systolic function, and causing an increase in cardiac pulsatile blood volume [69]. Shengmai Injection can regulate Toll-like receptor 4 (TLR4) and NF-*κ*B protein levels to inhibit inflammatory factors downstream of TLR4/NF-*κ*B signaling pathway, thereby improving cardiac dysfunction, reducing myocardial injury, and arresting heart failure in rats with dilated cardiomyopathy [70]. Xinmailong Injection inhibits the progression of heart failure by inhibiting ERK1/2, Akt/GSK3*β,* and GATA4 signaling pathways, reduces posterior left ventricular wall hypertrophy and increases left ventricular ejection fraction (LVEF) and left ventricular shortening (LVFS) [71]. It also effectively inhibits oxygen free radicals, stress response, improves cardiomyocyte protection, and reduces the cardiotoxicity of chemotherapeutic drugs [72]. Astragalus saponin contained in Huang qi injection can enhance myocardial contractility, dilate coronary arteries thus increasing myocardial blood supply, as well as improve myocardial cells' tolerance to hypoxia, protect myocardial cells from damage by inflammatory factors and free radicals, and improve cardiac function [73–75].

RETRACTED

Our sensitivity analysis showed that the overall results remained relatively stable when only studies with ≥80 cases were analyzed. The differences in LVEF between Shenfu injection and Shengmai injection, and in LVEDD among Huang qi injection, Xinmailong injection, and Shengmai injection may be due to the small number of studies on these outcomes. The overall results were relatively stable when ≥4 cycles of treatment were used as a condition for sensitivity analysis. Only the efficacy ranking of Xinmailong Injection and Shenqi fuzheng Injection was slightly different from the previous one, which may be related to the different number of patients included in these studies and the type of tumor included.

This Network Meta-analysis (NMA) took six CMIs as a starting point to analyze and compare their cardioprotective effects on patients after anthracycline treatment. It expands the therapeutic thinking on this type of disease and conveys the important value of CMIs in protecting patients' hearts, which is fully worthy of further promotion to countries outside China, where CMIs are not commonly used in Chinese medicine, becoming compatible and complementary to modern medicine, serving to broaden clinical diagnosis and treatment ideas, providing ideas for new drug development, and paying more attention to the cardiotoxicity of anthracyclines.

The use of CMIs to protect the hearts of patients on anthracycline chemotherapy is an excellent option, but challenges remain with this approach. Is it possible to specify the active therapeutic component in CMIs? Do these injections contain the same active ingredients or herbal monomers? Does it show differential treatment effects for different tumor patients? All of these issues are likely to be the subject of further research by CMIs in the future. However, these hypotheses should be more reliably substantiated by more in-depth basic research or higher quality clinical studies. We look forward to having more high-quality clinical studies in the future and using the NMA to make a greater contribution to the research of evidence-based Chinese medicine.

## 5. Limitations

There are some limitations to this study. ① The RCT studies included in this study did not specify the generation of random sequences, allocation concealment, blinding of investigators and subjects, and selective reporting of study results, which may have led to the presence of selection and measurement bias. ② There was some variation in the timing of CMIs among the included studies, including concomitant use with anthracyclines and use 3–5 d before the use of anthracyclines; therefore, the choice of the type of CMIs and the timing of the intervention may affect the discrimination of the results. ③ No safety indicators have been reported in the literature, so no conclusions can be drawn about the safety of CMIs. ④ The criteria for the type of tumor included in the study and the specific chemotherapeutic agents used were inconsistent, and the patients included were those with acute leukemia, breast cancer, stomach cancer, oesophageal cancer, ovarian cancer, malignant lymphoma, lung cancer, cervical cancer, etc.

RETRACTED

## 6. Conclusion

In this study, we evaluated six CMIs commonly used to combat cardiotoxicity of anthracycline-based chemotherapeutic agents in terms of different outcome indicators and summarized the efficacy of each CMI in terms of probability ranking. Network meta-analysis showed that Shenfu injection was associated with better LVEF values compared to chemotherapy only. Huang qi injection was most effective in improving the rate of ST-T segment (ECG change) alteration rates and CK-MB (U/L). Three CMIs (Shengmai Injection, Huang qi Injection and Xinmailong Injection) can significantly reduce LVEDD values. In a two-by-two comparison, Shengmai Injection was more effective than Huang qi Injection and Xinmailong Injection. Shenqi fuzheng Injection ranked highest in improving CK-MB (*μ*/L) (but not statistically significant). In summary, Huang qi Injection and Shenfu Injection performed better in all evaluation criteria. Shenmai Injection, Shenqi fuzheng Injection, Shengmai Injection, and Xinmailong Injection for the prevention and treatment of cardiac injury caused by anthracyclines, with different effects on different outcomes.

Although current studies have confirmed the unique advantages and efficacy of TCM in the prevention and treatment of anthracycline cardiotoxicity, the standardization, safety and efficacy of clinical application still require in-depth research. In the future, we look forward to strengthening the requirements for test methods. Distinguish between the type of tumor involved, the use of chemotherapeutic agents and the specific timing and dose of CMIs intervention. Completing higher-quality RCT studies, thus further validating the cardioprotective effects of CMIs in patients using anthracyclines, and making efforts for a more standardized and widespread use of CMIs.

RETRACTED

## Figures and Tables

**Figure 1:** Flowchart of study selection.

**Figure 2:** Results of risk of bias evaluation of included studies.

**Figure 3:** Reticulation of cardiotoxicity of anthracycline-based chemotherapeutic agents treated with CMI.

**Figure 4:** ST-T segment (ECG chenge).

**Figure 5:** Probability ranking of the effectiveness of six CMIs in improving the variability of the ST-T segment (ECG changes) of the ECG (A: chemotherapy only, B: Shenfu injection, C: Shenmai injection, D: Shenqi fuzheng injection, F: Shengmai injection, G: Xinmailong injection, H: Huang qi injection).

**Figure 6:** CK-MB-(U/L).

**Figure 7:** CK-MB-(*μ*g/L).

**Figure 8:** Probabilistic ranking of the effect of four measures on the improvement of CK-MB (U/L). (A: chemotherapy only, B: Shenfu injection, C: Shenmai injection, D: Shenqi fuzheng injection, F: Shengmai injection, H: Huang qi injection).

**Figure 9:** Probabilistic ranking of the improvement effect of three measures on CK-MB (*μ*/L). (A: chemotherapy only, B: Shenfu injection, C: Shenmai injection, D: Shenqi fuzheng injection, F: Shengmai injection, H: Huang qi injection).

**Figure 10:** LVEF.

**Figure 11:** Probability ranking of the effectiveness of five CMIs in LVEF. (A: chemotherapy only, B: Shenfu injection, D: Shenqi fuzheng injection, F: Shengmai injection, G: Xinmailong injection, H: Huang qi injection).

**Figure 12:** LVEDD.

**Figure 13:** Probability ranking of the effectiveness of four treatment measures in improving LVEDD. (A: chemotherapy only, D: Shenqi fuzheng injection, F: Shengmai injection, G: Xinmailong injection, H: Huang qi injection).

**Figure 14:** ST-T segment (ECG change) alteration rates forest plots.

**Figure 15:** CK-MB (U/L) and CK-MB (*μ*/L) forest plots.

**Figure 16:** LVEF forest plots.

**Figure 17:** LVEDD forest plots.

**Figure 18:** ST-T segment of ECG (ECG change) comparison-correction funnel chart.

**Figure 19:** LVEF comparison-correction funnel chart.

**Figure 20:** LVEDD comparison-correction funnel chart.

**Table 1:** Basic information on the six kinds of CMIs to be included.

Number	Generic name	Chemical composition	Botanical/animal name
1	Shenfu injection	Ginsenoside, aconitum alkaloids, inorganic salts, amino acids	Red Ginseng, monkshood
2	Shenmai injection	Ginsenoside, notoginsenoside, borneol glycoside, ophiopogonin homoisoflavonoids	Red Ginseng, *Ophiopogon japonicus*
3	Shenqi Fuzheng injection	Calycosin, Syringin, 5-Hydroxymethyl furfural, guanosine, vanillic acid	Codonopsis pilosula, *Astragalus membranaceus*
4	Shengmai injection	Fructose, flucose ginsenoside, excipient is polysorbate 80	Red Ginseng, *O. japonicus*, *Schisandra chinensis*
5	Xinmailong injection	Adenosine, protocatechuic acid, inosine,pyroglutamine dipeptide	*Periplaneta americana*
6	Huang qi injection	Formononetin, calycosin acetyl astragaloside I, astragaloside I	*A. membranaceus*

RETRACTED

**Table 2:** Characteristics of included studies.

Author	Sample (T/C)	Age (year)		Tumor type	Intervention		Time	Out-comes
		T	C		T	C		
Qu [37]	33/33	—	—	Breast cancer, stomach cancer, esophageal cancer, lung cancer, prostate cancer, ovarian cancer, cervical cancer, non-Hodgkinlymphoma	Shen fu injection°+°chemo-therapy	Chemo-therapy only	4∼6 cycles	(2)
Yang et al. [23]	50/46	—	—	Breast cancer, non-Hodgkinlymphoma	Shen fu injection°+°chemo-therapy	Chemo-therapy only	6 cycles	(1); (3)
Chen et al. [22]	47/45	31∼72 (58.25)	34∼73 (60.35)	Breast cancer, stomach cancer, esophageal cancer, malignant lymphoma	Shen fu injection°+°chemo-therapy	Chemo-therapy only	10∼14 d	(1); (2)
Shen [38]	80/80	53.74°±°8.84	54.45°±°9.23	Leukemia	Shen fu injection°+°chemo-therapy	Chemo-therapy only	6 cycles	(1); (2)
Wang et al. [24]	50/46	24∼66	28∼65	Breast cancer, cervical cancer, non-Hodgkinlymphoma	Shen mai injection°+°chemo-therapy	Chemo-therapy only	3 cycles	(1)
Ma [39]	50/50	—	—	Nonsmall cell lung cancer, breast cancer, cervical cancer, ovarian cancer, kidney cancer, prostate cancer, non-Hodgkinlymphoma	Shen mai injection°+°chemo-therapy	Chemo-therapy only	4∼6 cycles	(2)
Su [40]	35/30	23∼67	26∼65	Breast cancer, malignant lymphoma, stomach cancer, ovarian cancer	Shen mai injection°+°chemo-therapy	Chemo-therapy only	4∼6 cycles	(1)
Sun et al. [41]	42/41	—	—	Acute myelogenous leukemia	Shen mai injection°+°chemo-therapy	Chemo-therapy only	7 d	(1); (2)
Sun [42]	40/40	37.20°±°11.58	34.73°±°14.80	Acute myelogenous leukemia	Shen mai injection°+°chemo-therapy	Chemo-therapy only	7 d	(1); (2)
Chen [25]	45/41	—	—	Lung cancer, breast cancer, ovarian cancer, stomach cancer, non-Hodgkinlymphoma	Shen mai injection°+°chemo-therapy	Chemo-therapy only	7∼10 d	(1); (3)
Duan [43]	31/31	48°±°1.62	49°±°1.08	Malignant tumors (specific not available)	Shen qi fu zheng injection°+°chemo-therapy	Chemo-therapy only	28 d	(1)
Gu et al. [44]	40/40	—	—	Malignant lymphoma	Shen qi fu zheng injection°+°chemo-therapy	Chemo-therapy only	28 d	(1); (3)
Ning et al. [26]	28/26	42∼72	40∼74	Lung adenocarcinoma, squamous lung cancer, gastric adenocarcinoma, breast cancer, malignant lymphoma	Shen qi fu zheng injection°+°chemo-therapy	Chemo-therapy only	2∼4 cycles	(3)
Wang et al. [45]	60/60	—	—	Breast cancer, gastric cancer, lymphoma, esophageal cancer, soft tissue sarcoma, mediastinal tumor, small cell lung cancer, malignant tumor of unknown primary site	Shen qi fu zheng injection°+°chemo-therapy	Chemo-therapy only	6 cycles	(2); (3)
Wang et al. [27]	30/30	—	—	Breast cancer	Shen qi fu zheng injection°+°chemo-therapy	Chemo-therapy only	4 cycles	(1); (2); (3)
Wang [46]	30/31	56°±°16	55°±°13	Breast cancer, stomach cancer, ovarian cancer, non-Hodgkinlymphoma cervical cancer	Shen qi fu zheng injection°+°chemo-therapy	Chemo-therapy only	6 cycles	(1); (2); (3); (4)
Cui et al. [47]	22/20	—	—	Breast cancer	Shen qi fu zheng injection°+°chemo-therapy	Chemo-therapy only	4∼6 cycles	(1); (3)
Gong et al. [48]	28/30	—	—	Breast cancer	Shen qi fu zheng injection°+°chemo-therapy	Chemo-therapy only	2 treatment courses	(3); (4)
Chen [28]	30/30	42.93°±°9.67	45.73°±°9.28	Acute myeloid leukemia, acute lymphoblastic leukemia, multiple myeloma	Shen qi fu zheng injection°+°chemo-therapy	Chemo-therapy only	3 w	(1)
Cai et al. [49]	40/40	—	—	Breast cancer	Shen qi fu zheng injection°+°chemo-therapy	Chemo-therapy only	6 cycles	(1); (3)
Ding et al. [29]	22/26	—	—	Malignant tumors of the breast	Shen qi fu zheng injection/fu fang ku shen injection°+°chemo-therapy	Chemo-therapy only	4∼6 cycles	(1)
Zhang [50]	57/62	—	—	Breast cancer	Sheng mai injection°+°chemo-therapy	Chemo-therapy only	4 cycles	(1); (3); (4)
Wang et al. [36]	36/33	—	—	Breast cancer, ovarian cancer, stomach cancer, colon cancer	Sheng mai injection°+°chemo-therapy	Chemo-therapy only	14 d	(1); (3); (4)
Yan et al. [51]	112/104	—	—	Leukemia, non-Hodgkinlymphoma	Sheng mai injection°+°chemo-therapy	Chemo-therapy only	6 cycles	(1); (2); (3); (4)
Guo et al. [52]	43/43	43.8°±°6.5	45.5°±°6.2	Breast cancer, non-Hodgkinlymphoma, multiple myeloma	Sheng mai injection°+°chemo-therapy	Chemo-therapy only	2 w	(1)
He and Li [53]	40/40	51.5°±°3.5	51.3°±°3.4	Stomach cancer, breast cancer, ovarian cancer, malignant lymphoma	Xin mai long injection°+°chemo-therapy	Chemo-therapy only	6 cycles	(1); (3); (4)
Liu et al. [54]	29/28	61.7°±°5.9	58.7°±°6.1	Breast cancer, stomach cancer, ovarian cancer, malignant lymphoma	Xin mai long injection°+°chemo-therapy	Chemo-therapy only	6 cycles	(1); (3); (4)
Zou [55]	31/30	40°±°11	45°±°7	Breast cancer, malignant lymphoma, ovarian cancer, stomach cancer	Xin mai long injection°+°chemo-therapy	Chemo-therapy only	6 treat-ment courses	(1); (3); (4)
Wu et al. [56]	45/43	52.2°±°6.4	51.9°±°7.1	Malignant tumors (specific not available)	Xin mai long injection°+°chemo-therapy	Chemo-therapy only	3 cycles	(1); (3); (4)
Yang et al. [30]	50/50	18∼60	19∼60	Acute leukemia	Xin mai long injection°+°chemo-therapy	Chemo-therapy only	3 treat-ment courses	(1); (3); (4)
Zhou et al. [57]	30/28	45.6°±°6.4	44.8°±°5.8	Malignant lymphoma, breast cancer, lung cancer, stomach cancer, ovarian cancer	Huang qi injection°+°chemo-therapy	Chemo-therapy only	2 w	(1); (3); (4)
Yang and Dong [58]	30/31	25∼72	20∼71	Breast cancer, stomach cancer, ovarian cancer, non-Hodgkinlymphoma, cervical cancer	Huang qi injection°+°chemo-therapy	Chemo-therapy only	6 cycles	(1); (3); (4)
Li [59]	40/40	38.36°±°9.5	37.58°±°7.8	Breast cancer	Huang qi injection°+°chemo-therapy	Chemo-therapy only	6 cycles	(2); (3); (4)

ST-T segment (ECG changes) change rate; creatine kinase isoenzyme (CK-MB); left ventricular ejection fractions (LVEF) changes; ventricular ejection fractions (LVEF) changes; left ventricular end diastolic dimension (LVEDD).

RETRACTED

**Table 3:** ECG ST-T segment (ECG changes) variation network meta-analysis results.

Intervention	Chemotherapy only	Shenfu injection	Shenmai injection	Shenqifuzheng injection	Shengmai injection	Xinmailong injection	Huangqi injection
Chemotherapy only	1	—	—	—	—	—	—
Shenfu injection	6.50 (2.32, 19.37)	1	—	—	—	—	—
Shenmai injection	2.86 (0.83, 9.21)	0.44 (0.08, 2.06)	1	—	—	—	—
Shenqi Fuzheng injection	2.45 (1.18, 5.05)	0.38 (0.10, 1.30)	0.86 (0.22, 3.60)	1	—	—	—
Shengmai injection	3.11 (1.16, 8.92)	0.48 (0.11, 2.10)	1.09 (0.24, 5.74)	1.27 (0.39, 4.71)	1	—	—
Xinmailong injection	6.30 (2.44, 18.00)	0.98 (0.23, 4.39)	2.23 (0.49, 11.61)	2.57 (0.79, 9.45)	2.03 (0.51, 8.37)	1	—
Huang qi injection	6.42 (1.23, 43.07)	0.98 (0.14, 8.98)	2.27 (0.29, 22.69)	2.65 (0.44, 20.97)	2.05 (0.29, 16.70)	1.02 (0.14, 8.41)	—

**Table 4:** CK-MB network meta-analysis results.

Intervention	Chemotherapy only	Shenfu injection	Shenmai injection	Shenqi fuzheng injection	Shengmai injection	Huangqi injection
Chemotherapy only	1	0.15 (−5.97, 6.43)	0.07 (−3.50, 3.64)	2.71 (−1.89, 7.10)	—	—
Shenfu injection	20.46 (−20.21, 62.62)	1	−0.11 (−7.29, 6.95)	2.52 (−5.07, 9.96)	—	—
Shenmai injection	—	—	1	2.63 (−3.07, 8.34)	—	—
Shenqi Fuzheng injection	11.35 (−49.59, 72.62)	−8.98 (−81.29, 65.63)	—	1	—	—
Shengmai injection	37.19 (−20.08, 96.05)	17.06 (−53.59, 89.79)	—	25.94 (−60.48, 110.86)	—	—
Huangqi injection	44.01 (−15.69, 103.00)	22.94 (−48.66, 93.68)	—	32.47 (−52.41, 117.14)	7.00 (−76.87, 90.39)	1

U/L is the bottom left of the assay unit; ng/ml (*μ*g/L) is the top right of the assay unit; —: missing literature for comparison.

**Table 5:** LVEF network meta-analysis results.

Intervention	Chemotherapy Only	Shenfu injection	Shenqi Fuzheng injection	Shengmai injection	Xinmailong injection	Huangqi injection
Chemotherapy only	1	—	—	—	—	—
Shenfu injection	−10.51 (−20.36, −0.39)	1	—	—	—	—
Shenqi fuzheng injection	−4.75 (−7.63, −1.82)	5.75 (−4.67, 16.13)	1	—	—	—
Shengmai injection	−4.11 (−8.35, 0.24)	6.41 (−4.24, 17.37)	0.64 (−4.52, 5.87)	1	—	—
Xinmailong injection	−2.81 (−6.21, 0.63)	7.72 (−3.02, 18.12)	1.93 (−2.51, 6.32)	1.30 (−4.15, 6.64)	1	—
Huangqi injection	−6.48 (−12.68, 0.18)	4.12 (−7.46, 16.26)	−1.68 (−8.69, 5.71)	−2.34 (−9.89, 5.64)	−3.66 (−10.77, 4.07)	1

RETRACTED

**Table 6:** LVEDD network meta-analysis results.

Intervention	Chemotherapy only	Shenqi Fuzheng injection	Shengmai injection	Xinmailong injection	Hangqi injection
Chemotherapy only	1	—	—	—	—
Shenqi Fuzheng injection	3.59 (−1.36, 8.69)	1	—	—	—
Shengmai injection	7.97 (3.10, 12.99)	4.39 (−2.86, 11.44)	1	—	—
Xinmailong injection	4.78 (1.44, 7.95)	1.21 (−4.92, 6.94)	−3.18 (−9.37, 2.66)	1	—
Hangqi injection	7.87 (3.79, 12.05)	4.30 (−2.35, 10.71)	−0.11 (−6.51, 6.54)	3.09 (−2.05, 8.36)	1

**Table 7:** Sensitivity analysis (case number ≥80) ECG ST-T segment (ECG changes) variation network meta-analysis results.

Intervention	Chemotherapy only	Shen fu injection	Shen mai injection	Shenqi fuzheng injection	Sheng mai injection	Xin mai long injection
Chemotherapy only	1	—	—	—	—	—
Shenfu injection	8.63 (1.36, 56.63)	1	—	—	—	—
Shenmai injection	3.09 (0.54, 16.23)	0.36 (0.03, 4.34)	1	—	—	—
Shenqi Fuzheng injection	3.16 (0.15, 64.81)	0.38 (0.01, 12.09)	1.03 (0.03, 34.79)	1	—	—
Shengmai injection	3.20 (0.58, 21.69)	0.37 (0.03, 5.75)	1.05 (0.10, 13.46)	1.00 (0.03, 37.53)	1	—
Xinmailong injection	5.11 (0.79, 58.13)	0.60 (0.04, 14.14)	1.67 (0.14, 32.95)	1.00 (0.03, 37.54)	1.59 (0.11, 32.68)	1

**Table 8:** Sensitivity analysis (case number ≥ 80) CK-MB network meta-analysis results.

Intervention	Chemotherapy only	Shenfu injection	Shenmai injection	Shenqi Fuzheng injection	Shengmai injection	Huangqi injection
Chemotherapy only	—	—	0.08 (−0.19, 0.36)	—	—	—
Shenfu injection	20.86 (−20.46, 61.41)	1	—	—	—	—
Shenmai injection	—	—	1	—	—	—
Shenqi Fuzheng injection	11.58 (−47.05, 70.19)	−9.18 (−79.74, 61.62)	—	1	—	—
Shengmai injection	37.50 (−21.42, 96.56)	16.42 (−56.85, 87.98)	—	26.15 (−59.14, 108.67)	1	—
Huangqi injection	43.97 (−13.37, 102.06)	22.82 (−48.31, 94.70)	—	32.37 (−50.89, 114.68)	6.22 (−77.01, 91.46)	1

U/L is the bottom left of the assay unit; ng/ml (*μ*g/L) is the top right of the assay unit; —: missing literature for comparison.

**Table 9:** Sensitivity analysis (case number ≥ 80) LVEF network meta-analysis results.

Intervention	Chemotherapy only	Shenfu injection	Shenqi fuzheng injection	Shengmai injection	Xinmailong injection	Huangqi injection
Chemotherapy only	1	—	—	—	—	—
Shenfu injection	−10.31 (−22.05, 1.49)	1	—	—	—	—
Shenqi Fuzheng injection	−9.30 (−16.51, −2.20)	1.01 (−12.94, 14.91)	1	—	—	—
Shengmai injection	−3.28 (−10.36, 4.34)	7.08 (−6.50, 21.00)	6.04 (−4.01, 16.51)	1	—	—
Xinmailong injection	−2.41 (−8.21, 3.40)	7.90 (−5.01, 20.80)	6.90 (−2.32, 16.00)	0.89 (−8.65, 10.01)	1	—
Huangqi injection	−7.6 (−18.26, 2.40)	2.61 (−13.53, 18.44)	1.65 (−11.23, 14.18)	−4.40 (−17.73, 8.08)	−5.24 (−17.55, 6.46)	1

RETRACTED

**Table 10:** Sensitivity analysis (case number ≥ 80) LVEDD network meta-analysis results.

Intervention	Chemotherapy only	Shengmai injection	Xinmailong injection	Hangqi injection
Chemotherapy only	1	—	—	—
Shengmai injection	7.88 (−0.08, 15.46)	1	—	—
Xinmailong injection	5.57 (−0.06, 10.91)	−2.23 (−11.73, 7.28)	1	—
Hangqi injection	6.39 (−1.38, 14.30)	−1.49 (−12.14, 10.01)	0.84 (−9.05, 10.34)	1

**Table 11:** Sensitivity analysis (intervention ≥4 cycles) ECG ST-T segment (ECG changes) variation network meta-analysis results.

Intervention	Chemotherapy only	Shenfu injection	Shenmai injection	Shenqi fuzheng injection	Shengmai injection	Xinmailong injection	Huangqi injection
Chemotherapy only	1	—	—	—	—	—	—
Shenfu injection	4.63 (0.69, 37.37)	1	—	—	—	—	—
Shenmai injection	2.91 (0.15, 67.18)	0.62 (0.02, 23.05)	1	—	—	—	—
Shenqi fuzheng injection	2.97 (0.90, 9.98)	0.63 (0.06, 5.94)	1.01 (0.03, 23.86)	1	—	—	—
Shengmai injection	1.95 (0.36, 15.30)	0.41 (0.03, 7.03)	0.67 (0.02, 25.15)	0.66 (0.08, 7.58)	1	—	—
Xinmailong injection	11.87 (2.28, 77.13)	2.54 (0.19, 38.12)	3.99 (0.12, 162.46)	4.03 (0.50, 38.08)	6.04 (0.47, 72.04)	1	—
Huangqi injection	4.86 (0.29, 102.92)	1.02 (0.03, 35.61)	1.69 (0.03, 106.26)	1.61 (0.08, 44.33)	2.46 (0.07, 74.66)	0.41 (0.01, 12.77)	1

**Table 12:** Sensitivity analysis (intervention ≥4 cycles) CK-MB network meta-analysis results.

Intervention	Chemotherapy only	Shenfu injection	Shenmai injection	Shenqi fuzheng injection	Shengmai injection	Huangqi injection
Chemotherapy only	1	0.20 (−2.98, 3.45)	0.36 (−2.77, 3.57)	1.21 (−1.08, 3.51)	—	—
Shenfu injection	37.83 (−18.42, 92.02)	1	0.14 (−4.45, 4.74)	1.00 (−2.89, 4.99)	—	—
Shenmai injection	—	—	1	0.89 (−3.11, 4.77)	—	—
Shenqi Fuzheng injection	11.63 (−44.36, 66.55)	−26.52 (−102.27, 52.49)	—	1	—	—
Shengmai injection	37.32 (−16.62, 92.07)	−0.54 (−73.56, 77.65)	—	25.95 (−51.34, 103.14)	1	—
Huangqi injection	43.62 (−11.31, 98.10)	5.62 (−72.10, 82.72)	—	32.20 (−44.66, 108.95)	6.42 (−70.85, 84.33)	1

U/L is the bottom left of the assay unit; ng/ml (*μ*g/L) is the top right of the assay unit; —: missing literature for comparison.

**Table 13:** Sensitivity analysis (intervention ≥ 4 cycles) LVEF network meta-analysis results.

Intervention	Chemotherapy only	Shenfu injection	Shenqi fuzheng injection	Shengmai injection	Xinmailong injection	Huangqi injection
Chemotherapy only	1	—	—	—	—	—
Shenfu injection	−10.56 (−19.04, −1.68)	1	—	—	—	—
Shenqi Fuzheng injection	−4.04 (−6.96, −1.37)	6.46 (−2.75, 15.34)	1	—	—	—
Shengmai injection	−3.50 (−7.31, 0.61)	7.05 (−2.56, 16.54)	0.54 (−4.07, 5.56)	1	—	—
Xinmailong injection	−3.87 (−7.13, −0.30)	6.68 (−2.72, 15.83)	0.15 (−4.17, 4.83)	−0.36 (−5.63, 4.72)	1	—
Huangqi injection	−6.76 (−12.70, −0.42)	3.78 (−6.64, 14.38)	−2.73 (−9.13, 4.30)	−3.32 (−10.35, 4.07)	−2.91 (−9.66, 4.15)	1

RETRACTED

**Table 14:** Sensitivity analysis (intervention ≥ 4 cycles) LVEDD network meta-analysis results.

Intervention	Chemotherapy only	Shenqi Fuzheng injection	Shengmai injection	Xinmailong injection	Hangqi injection
Chemotherapy only	1	—	—	—	—
Shenqi Fuzheng injection	8.72 (0.61, 16.77)	1	—	—	—
Shengmai injection	7.79 (0.35, 15.40)	−0.90 (−11.89, 10.25)	1	—	—
Xinmailong injection	4.72 (0.00, 9.09)	−4.02 (−13.42, 5.11)	−3.03 (−12.17, 5.76)	1	—
Hangqi injection	7.42 (1.85, 13.29)	−1.25 (−11.00, 8.73)	−0.41 (−9.59, 9.11)	2.76 (−4.16, 10.20)	1

## Abbreviations

TCM: Traditional Chinese medicine
CMI: Chinese medicine injection
RCTs: Randomized controlled trials
NMA: Network meta-analysis
cTnI: Cardiac troponin I
CK-MB: Creatine kinase isoenzymes MB
LVEF: Left ventricular ejection fraction
LVEDD: Left ventricular end-diastolic internal diameter
SUCRA: The surface under the cumulative ranking curve
FDA: U.S. Food and drug administration
EMA: European drug administration
LVFS: Left ventricular fractional shortening.
